# Image Processing for mHealth-Based Approach to Detect the Local Tissue Inflammation in Cutaneous Leishmaniasis: A Proof of Concept Study

**DOI:** 10.1155/2021/4208254

**Published:** 2021-11-27

**Authors:** Hermali Silva, Kalaivani Chellappan, Nadira Karunaweera

**Affiliations:** ^1^Department of Parasitology, Faculty of Medicine, University of Colombo, Colombo, Sri Lanka; ^2^Department of Electrical, Electronic & Systems Engineering, Faculty of Engineering & Built Environment, National University of Malaysia, Bangi, Selangor, Malaysia

## Abstract

Skin lesions are a feature of many diseases including cutaneous leishmaniasis (CL). Ulcerative lesions are a common manifestation of CL. Response to treatment in such lesions is judged through the assessment of the healing process by regular clinical observations, which remains a challenge for the clinician, health system, and the patient in leishmaniasis endemic countries. In this study, image processing was initially done using 40 CL lesion color images that were captured using a mobile phone camera, to establish a technique to extract features from the image which could be related to the clinical status of the lesion. The identified techniques were further developed, and ten ulcer images were analyzed to detect the extent of inflammatory response and/or signs of healing using pattern recognition of inflammatory tissue captured in the image. The images were preprocessed at the outset, and the quality was improved using the CIE *L*∗*a*∗*b* color space technique. Furthermore, features were extracted using the principal component analysis and profiled using the signal spectrogram technique. This study has established an adaptive thresholding technique ranging between 35 and 200 to profile the skin lesion images using signal spectrogram plotted using Signal Analyzer in MATLAB. The outcome indicates its potential utility in visualizing and assessing inflammatory tissue response in a CL ulcer. This approach is expected to be developed further to a mHealth-based prediction algorithm to enable remote monitoring of treatment response of cutaneous leishmaniasis.

## 1. Introduction

Interdisciplinary approaches are becoming increasingly popular in the health sector, specially to improve the diagnosis and management of various diseases [1–4]. Variety of methods of image processing and analyses are available for extracting valuable information from raw images taken from cameras [5]. With the advent of mobile phones, the concept of mobile health or mHealth emerged and it could be broadly described as a medical and public health practice supported by mobile devices such as mobile phones [6]. With the increased usage of smart phones and tablets among people, their contribution to image analysis applications and mHealth has also been noteworthy [7].

Leishmaniasis is a neglected tropical disease affecting about 88 countries mainly in the tropics and subtropics (http://www.cdc.gov). A bite of an infected sand fly can cause the disease in humans, and the type of disease manifestations may vary from localized lesions or ‘wounds' on skin to visceral form which affects the internal organs of the patient. The most common disease form in the world is cutaneous leishmaniasis (CL) which affects the skin [8]. According to their morphological appearance, CL lesions are commonly categorized as papules, nodules, plaques, and ulcers. Of these, the most common is ulcers [8]. A CL ulcer has a ‘volcanic' appearance with a central crater and a raised border [9].

Visual and clinical assessment of the lesions is generally used in CL for monitoring the treatment response. This requires a skilled, trained medical personnel. However, some of the regions burdened with leishmaniasis are remote where mobility and access to specialized dermatology treatment centres and specialized medical personnel are limited. Even in areas with access to the above, some patients may opt to seek follow-up through mHealth due to the convenience, economic reasons, or when movements are restricted such as during the current COVID-19 pandemic. Furthermore, accessibility to mobile devices even in tropical countries, including Sri Lanka has exponentially increased during the past decade. A series of surveys on the access and use of information and communications technology, conducted from 2017 to 2019, found that most of the Asian countries surveyed had about two-thirds of their 15–65-year-old population owning a mobile phone, with 78% to be exact in Sri Lanka [10]. This survey furthermore identified that Sri Lankan rural dwellers had a similar likelihood of owning a mobile phone as the urban dwellers. The need to seek digitalized solutions for health-related issues that may be accessed remotely is felt stronger now than ever due to the ‘new normal' adaptations required to survive the pandemic situation.

mHealth approaches using mobile phone applications for presumptive diagnosis of leishmaniasis and using image processing for assessment of skin lesions have been reported with emphases on the need and space for further improvement [11–14]. Various image processing techniques are employed at different stages of conversion of a raw image (*viz* image acquisition, image preprocessing, clustering, and classification), into making it more useful for extracting information [15]. Techniques such as color space, principal component analysis (PCA), and pattern recognition have been used for image processing in various medical fields [16–18].

Studies have shown the presence of a local inflammatory reaction at the lesion site in CL [19, 20]. This inflammatory response includes increased vascular permeability, dilatation of blood vessels in the dermis, and infiltration of the lesion site with immune cells, which would contribute to the swelling and the morphology of the lesion [13]. Even though the inflammatory changes are not pathognomonic to CL, the reduction in the inflammatory response is an indication of healing or a good response to treatment in CL. While utilizing microscopy and other parasitological laboratory methods to confirm the diagnosis of leishmaniasis, a technique to visualize the inflamed tissue in a CL lesion will be valuable in treatment monitoring and follow-up of patients. Appreciating the mHealth concept, in the simplest scenario, the patients or the primary health care workers can capture the lesion image using a mobile phone and upload to a cloud based diagnostic centre for an analysis report to be forwarded to a consultant medical specialists for treatment monitoring and evaluation purposes as part of clinical management.

Based on the currently available information in digital and health fields, the authors hypothesized that image processing could be used to visualize the inflammatory tissue in the CL lesions and could be utilized as a noncontact assessment or a self-assessment method to detect the inflammatory response in CL. Thus, the aim of this study was to investigate the concept of using image processing and analysis techniques to process mobile captured JPEG images of cutaneous leishmaniasis lesions to detect the inflamed tissue and relating it to the treatment response of the lesions.

## 2. Materials and Methods

### 2.1. Patients and Image Acquisition

Fifty patients who attended the District General Hospital, Hambantota, Sri Lanka, for treatment of cutaneous leishmaniasis were selected for this study. Parasitological confirmation of leishmaniasis was made by microscopy and/or culture. Color images of the lesions were taken from a mobile phone, before starting the treatment with weekly injections of intralesional sodium stibogluconate (IL-SSG), which is an antimony containing drug used as the standard treatment for CL in Sri Lanka [21]. A preliminary image processing was done for 40 images which included all phenotypes (papules *n* = 10, nodules *n* = 10, plaques *n* = 10, and ulcers n =10) as given below under section (A), to establish an image processing technique to extract features from the images which could be related to the inflammatory response and/or treatment response of all types of CL lesions. Since it was noted through the results of the preliminary analysis that the areas with the inflamed tissue in ulcers could be visualized differently and clearly from the healthy tissue, the image processing methodology was further developed into an agile integration methodology of eight blocks to detect the extent of inflammatory response and/or signs of healing in ulcers, using 10 images of ulcers (Section (B)). Ethical approval for this study was obtained from the Ethics Review Committee (EC/16/080), Faculty of Medicine, University of Colombo (http://www.med.cmb.ac.lk), Sri Lanka.

- Preliminary image processing (*n* = 40, phenotypes: papules, nodules, plaques, ulcers)

An image processing technique using MATLAB (The MathWorks, Inc., Natick, Massachusetts, United States) was adapted to process 40 mobile captured JPEG images. The images were resized to 256 × 256 pixel resolution, and grayscale conversion was done to standardize the variation of images. The standardized images were enhanced by using a contrast stretching algorithm to identify the boundary of the lesion to be cropped. The cropped images were further processed through thresholding and contour analysis, to cluster between poor responders and those who were sensitive to treatment with IL-SSG injections as defined earlier [22]. Briefly, ‘sensitive/cured' was defined as lesions clinically completely healed (as per previously used criteria) following 10 or lesser number of IL-SSG weekly injections and ‘poor response' means lesions that failed to completely heal by 10 IL-SSG weekly injections. The variance of images was studied to confirm the contour analysis outcome. Findings were compared with the treatment response.

(B) Further image processing to establish a technique for inflammation detection in ulcers (*n* = 10)

### 2.2. Image processing technique

An agile integration methodology in which microprocesses can be added or removed without affecting the macro processing of the images was used. This methodology was built on eight blocks that were attachable and detachable as per the requirement of image analysis and the clinical reporting needs.  Figure 1 represents the system block diagram of the implemented technique of image processing with eight different blocks.

### 2.3. Image preperation

Included the execution of the first two blocks (i.e., RGB image capture and cropping) of Figure 1. The selected images for this study were captured from a mobile phone and were in Joint Photographic Experts Group (JPEG) format. These RGB images contained elements less relevant to the ulcer, such as the ruler and background components. Thus, the raw images in the RGB color space were cropped to a width to height ratio of one, in order to reduce the unnecessary pixels in the image and to focus on the skin lesion [23]. A manually cropped image was processed using edge detection algorithm which determined the centre of the ulcer and expanded proportionally to the edge of the ulcer to identify the boundaries [24]. Sharp discontinuities in the image caused by sudden variations in the pixel intensity are recognized by the edge detection algorithm to establish the ulcer boundaries [24, 25].

### 2.4. Image preprocessing

Color space transformation is a significant step in preprocessing digital images. A color space describes colors numerically and is defined as a mathematical model which represents a color by three or four color components [26]. By converting the color images of the skin lesions to a color space, enhancement of both the elements of interest and the wide range of skin colors could be achieved [27]. This was achieved in the current study by executing the third block in Figure 1, by transforming the cropped RGB image into the CIE 1976 *L*∗*a*∗*b* color space (CIELAB). The CIELAB is a color space system which can distinguish colors from lightness/illumination; it is device-independent, covers the entire range of human daylight color perception or the gamut, and results in a saturated intensity value. Thus, CEILAB was used for further processing of the cropped image to intensify the cropped *RGB* image pixel values to make them become darker or lighter corresponding to different areas on the skin with related clinical manifestations.

### 2.5. Image segmentation

The luminosity channel was extracted from the CIELAB color space and the resultant saturated image was further enhanced by using the PCA to convert it to grayscale. PCA reduces dimensionality while minimizing information loss and increasing the capture of important information in the images [28]. PCA is a dimensionality reduction technique that can be used to solve object recognition problems. The dimensionality reduction benefits in avoiding voluminous calculations and is robust to the noise in the images. PCA transforms the original image data into a subspace set of principal components, of which the first principal component captures the greatest amount of variance among the images, while the second principal component provides the vector of the directions orthogonal to the first principal component.

In this study, the dimension of the image was given by the square image of size *x* × *y* in pixels, represented by a *x* × *y* matrix. The mean of every dimension of the whole dataset was calculated, and the covariance matrix of the two variables *x* and *y* was calculated by the equation (1). Eigenvalues and eigenvectors were obtained from the covariance matrix [29]. The eigenvalues were then sorted in to descending order to give the components in the order of significance. Eigenvectors with small eigenvalues were removed by the filter, and the eigenvectors with the largest eigenvalues were chosen to transform the dataset into a new subspace.

(1) $$\begin{array}{c} \text{Cov}\left(X,Y\right)=\frac{1}{n-1}\overset{n}{\underset{i=1}{\sum }}\left(Xi-\underline{x}\right)\left(Yi-\underline{y}\right). \end{array}$$

By image preprocessing and segmentation steps, pixels of the ulcers were separated from the background pixels that made way for the inner tissues of the ulcers to be analyzed.

### 2.6. Image analysis

This is the extraction of meaningful information from images corresponding to the 6^th^ and 7^th^ blocks in Figure 1. Based on the PCA grayscale image, a histogram was drawn to represent the pixel values (*x* axis: from 0 to 255) and their corresponding frequencies (*y* axis) in the image. The histogram shape thresholding technique was used for the ulcer region determination. This technique was applied indicating that images acquired following the acquisition protocol mentioned above resulted in a histogram with single peak, as shown in the results (Figure 2). The histogram shape thresholding requires finding the optimum threshold to separate the background (dark) from the foreground (bright) [30]. In a histogram representation of an image, there will be two regions that indicate the presence of dark and bright objects [30]. The optimum threshold was calculated using the quantile regression method which allows understanding relationships between variables outside of the mean of the data, making it useful to understand the outcomes that are not normally distributed and that have a nonlinear relationship with the predictor variables. Hence, the threshold value for this study was identified to be between 35 and 200 as it was found to be suitable for reducing the amount of excessive darkness or brightness in the image as shown in the results (Figure 2).

### 2.7. Pattern recognition

The final block of the method was performed using the Signal Processing Toolbox in MATLAB (MATLAB 2017b, The MathWorks, Inc., Natick, Massachusetts, United States) to complete the pattern recognition process by providing a function to analyze, preprocess, and extract features of the signals. The Signal Analyzer application in the toolbox facilitated the visualization, measurement, and analyzation of the signals (MATLAB 2020a, The MathWorks, Inc., Natick, Massachusetts, United States). The pixel values ranging from 35 to 200 were displayed in the time domain followed by the visual representation of the variation in frequency and time of the image using the signal spectrogram. The pattern recognition process was completed by conducting the analysis on the signal spectrogram. In brief, the pixel values of the image were read into the workspace of the Signal Analyzer in MATLAB. The application was used to plot the extracted information and to display the pattern distribution using a spectrogram. The data analysis was done based on the spectrogram obtained.

## 3. Results and Discussion

- Preliminary image processing (*n* = 40)

In thresholding analysis (Figures 3(b), 3(e), 3(h), and 3(k)), images following thresholding showed lesion areas with active inflammation in white and healthy tissue in black. There was a ‘scattered' appearance of white and black areas, indicating a nonhomogeneous localization of inflamed tissue and healthy tissue, prior to starting treatment in the lesions cured with IL-SSG (Figures 3(b) and 3(e)). However, the treatment failed lesions had homogenous regions of inflammation in the pretreatment stage (Figures 3(h) and 3(k) ).

In contour analysis (Figures 3(c), 3(f), 3(i), and 3(l)), active contour images show consistent color representation in the lesion area (Figures 3(i) and 3(l)) prior to treatment in the treatment failed category of lesions.

Variance (Figure 4) of the pixels of the image was calculated by MATLAB, to confirm the contour analysis outcome of the color consistency. Treatment failed lesions had lower variance (i.e., pixel intensities were closer to the mean) value which confirms the consistent color representation.

Thresholding, contour analysis, and variance were able to detect lesions with high inflammation. Thresholding and contour analyses of pretreatment images could differentiate IL-SSG treatment failures from those who got cured, with a 52.5% accuracy. Since a color pattern distribution in the inflamed region was observed through this preliminary image processing, the techniques were further developed to detect inflammation in the ulcers.

(B) Further image processing to detect inflammation in ulcers (*n* = 10)

In image preparation, Figure 5 shows the acquired raw RGB image and the resultant image after a self-customized cropping algorithm was applied, for three ulcers. The cropping algorithm significantly removed nonessential components and background elements from the ulcer image. Images were cropped to a width to height ratio of 1 to standardize the aspect ratio of the image to reduce the unwanted area around the lesion.

In image preprocessing and image segmentation, processed images obtained after luminosity extraction and PCA of the luminosity images obtained from color space transformation of the cropped RBG images are shown in Figure 6. Features concealed in previous images can be seen more clearly in the PCA-based grayscale images.

In image analysis, histograms were drawn based on the grayscale images to represent the pixel values and their corresponding frequency in the image (Figures 2(a)–2(c)). Thresholding was performed on the image to extract the information for ulcer profiling. Best thresholding which minimized the excess darkness or lightness for this study was found to be between 35 and 200. Figures 2(d)–2(f) show the histograms based on the images after thresholding was applied. Figures 2(g)–2(i) represent the threshold image after applying the threshold value range of 35 to 200. When the threshold value is applied to the image, the intensity values outside the selected range gets converted to the color black represented by 0, whereas the pixel values in the range are used for the analysis of the image.

In pattern recognition, the color pattern distribution was illustrated as in Figure 7. The yellow regions in the spectrogram represented the inflamed issue, while the dark blue regions were the healthy or healed tissue.

The image obtained after applying thresholding was translated to a signal based on the pixel distribution to recognize patterns, and the extracted information was plotted in MATLAB and the pattern distribution was displayed using a signal spectrogram (Figure 8).

Differences between the completely cured and treatment failed lesions were observed when the 40 pretreatment images were analyzed using thresholding and contour analyses. The ‘scattered' appearance of white and black areas, indicating a nonhomogeneous localization of inflamed tissue, and the consistent color representation in the lesion area were seen in lesions that ultimately failed treatment with IL-SSG. However, the study of the variances indicated that the accuracy of this prediction was 52.5%. Inclusion of different clinical types, demographic differences of the host, and variable time periods since the onset to capturing of the lesion images may be viewed as limitations of this analysis, which would have resulted in low accuracy. This analysis is promising as an antimony resistance predictor and warrants further studies targeting clinical phenotypes separately. However, when only ulcers were further analyzed, the image processing technique (Figure 1) used resulted in the possibility of inflammation profiling of the ulcer. However, this method of image processing can be also used to evaluate the process of inflammation in nonleishmaniasis lesions and, therefore, is not specific to the CL ulcers. The lack of specificity for leishmaniasis may be viewed as a limitation. However, this approach is still valuable for assessing the reduction of inflammation as an indication of healing in skin lesions as tested and confirmed in this study using leishmaniasis patients whose diagnosis was confirmed through laboratory testing. The color pattern in the spectrograms can assist the clinician to assess the healing of the lesions and the response to treatment through digital visualization of the tissue changes due to inflammation in the lesion. This will aid the clinician specially when the fine capturing of tissue changes may sometimes be masked during direct clinical observations mostly by the surrounding healing tissues. Such obstacles could be overcome by this image processing technique. Furthermore, in a remote set up or when a clinician is not easily accessible, a patient can be instructed to take a photograph of the lesion using his mobile phone and that could be accessed remotely by trained personnel to aid in patient management. Since the technique demonstrated in this study is likely to be applicable for any image and independent from the device from which they were captured, it is an added advantage in a mHealth approach.

## 4. Conclusions

The study demonstrates the potential utility of pattern recognition technique based on image analysis of skin ulcers that capture the extent of inflammatory tissue on the surface. The advantages of further development of the technique and its use in clinical practice will include cost saving and relieving patients from suffering undue stress of repeated hospital visits that are required during the follow-up period of antileishmania therapy in CL for clinical monitoring purposes. Studies are continued to analyze larger numbers of pretreatment CL skin lesion color images to develop a mHealth-based prediction algorithm for antimony response for cutaneous leishmaniasis. In conclusion, the mHealth approach assisted by image processing techniques and cloud based storage, analysis, and reporting may aid in the remote monitoring of cutaneous leishmaniasis ulcers and development of mHealth-based prediction algorithm for antimony response in cutaneous leishmaniasis.

## Figures and Tables

**Figure 1:** System block diagram of the agile integration technique for image processing and analysis.

**Figure 2:** Image analysis. (a–c) Histograms before thresholding. (d–f) Histograms after thresholding. (g–i) Images after applying thresholding.

**Figure 3:** Thresholding and contour analyses of leishmaniasis lesions.

**Figure 4:** Variance in the images of the IL-SSG sensitive and poorly responded lesions.

**Figure 5:** Image preparation–application of cropping algorithm to the raw RBG images taken from a smart phone.

**Figure 6:** Image preprocessing and image segmentation. (a–c) Luminosity image obtained from color space transformation of the cropped RBG image. (d–f) Corresponding grayscale images obtained after luminosity extraction and principal component analysis.

**Figure 7:** Color pattern distribution.

**Figure 8:** Signal spectrogram of the 10 ulcer images.

## Data Availability

All the data supporting the conclusions are within the manuscript.
